RETRACTED

# Structure based sequence analysis & epitope prediction of gp41 HIV1 envelope glycoprotein isolated in Pakistan

**DOI:** 10.1186/1479-0556-10-4

**Published:** 2012-06-20

**Authors:** Syyada Samra Jafri, Saliha Kiran, Syed Babar Jamal, Masaud Shah

**Affiliations:** 1 University of the Punjab, Lahore, Pakistan; 2 Government College University, Faisalabad, Pakistan; 3 International Islamic University Islamabad, Islamabad, Pakistan

**Keywords:** Human immunodeficiency virus, Pakistan, gp41, Epitopes, Bioinformatics

## Abstract

**Background:**

Gp41 is an envelope glycoprotein of human immune deficiency virus (HIV). HIV viral glycoprotein gp41, present in complex with gp120, assists the viral entry into host cell. Over eighty thousands individuals are HIV infected in Pakistan which makes about 0.2% of 38.6 million infected patients worldwide. Hence, HIV gp41 protein sequences isolated in Pakistan were analyzed for the CD4 and CD8 T cells binding epitopes.

**Results:**

Immunoinformatics tools were applied for the study of variant region of HIV gp41envelope protein. The protein nature was analyzed using freely accessible computational software. About 90 gp41 sequences of Pakistani origin were aligned and variable and conserved regions were found. Four segments were found to be conserved in gp41 viral protein. A method was developed, involving the secondary structure, surface accessibility, hydrophobicity, antigenicity and molecular docking for the prediction and location of epitopes in the viral glycoprotein. Some highly conserved CD4 and CD8 binding epitopes were also found using multiple parameters. The predicted continuous epitopes mostly fall in the conserved region of 1–12; 14–22 and 25–46 and can be used as effective vaccine candidates.

**Conclusions:**

The study revealed potential HIV subtype a derived cytotoxic T cell (CTL) epitopes from viral proteome of Pakistani origin. The conserved epitopes are very useful for the diagnosis of the HIV 1 subtype a. This study will also help scientists to promote research for vaccine development against HIV 1 subtype a, isolated in Pakistan.

## Introduction

An envelope virus HIV-1 expresses a surface glycoprotein mediating the attachment and fusion of virus with cellular membranes. HIV carries nearly 70 spikes [1] and is transmitted through mucosal secretions during sexual intercourse. CD4^+^T cells present in lymphoid organs and blood is the main site of infection.

During mid-1990s, first X-Ray crystal structure of GP-41 was solved. GP-41 mediates fusion of target cells to HIV-1. Understanding of its structure provides the understanding of virus entry into the host and describes the mode of action of compounds that block this process. As the infection cycle is initiated by the fusion of viral proteins with cell membranes, followed by the release of viral genome and proteins into the host. HIV-1 follows a multi-step process to enter into the host. This multi-step entry process provides active targets for the development of new therapeutic agents to block this entry. Designing of specific agents which can create hindrance in the entry of viral protein at each step are of considerable importance and substantial progress has been made in understanding the entry of HIV in host cell.

RETRACTED

GP-41 interacts with GP-120 non-covalently forming an oligomeric structure. Crystallographic and physical data suggests trimeric GP-41 – Gp-120)_3_ form of this oligomeric structure. It is postulated that GP-41 facilitates the fusion of viral cell membrane with the target’s membrane and undergoes major conformational rearrangements in a “spring-loaded mechanism” elaborated for influenza hemagglutinin [2]. HIV-1 is thought to be the major cause of infection in Pakistan. A core is present in the “sprung” conformation of GP-41[3,4] which is formed by an extended triple-stranded α-helical coiled coil. Outside of the coil is packed in reverse direction by carboxy-terminal α-helix bringing carboxy and amino terminals close to each other at long rod end. It is found that GP-41 is in stable state in the form of sprung conformation. Vaccine designing is a complicated process in envelop proteins due to the presence of several forms with distinct conformations. Mature oligomer may not have most of the epitopes on unprocessed oligomeric or monomeric envelop molecule.

## Materials and methods

### Sequences searching

NCBI protein database was used for the retrieval of gp 41, HIV1 subtype a proteins sequences of. 194 aa sequences were selected out of 200 retrieved from database in FASTA format.

### Alignment and conservancy

Multiple alignment of sequences and conservancy was found using offline ClastralW tool [5] useful for large no of sequences.

### T-cell epitopes of HIV gp41 protein prediction

Selected sequences were used for T-Cell epitope mapping using Epijen online software. A*0201, A*0301, A*1101 and B*07 were four HLA alleles used for predicting epitopes which have been reported to be recognize in more than 90% of the world population, regardless of ethnicity.

### Secondary structure prediction

SOPMA library [6], which is freely available server, was used for secondary structure prediction (http://npsa-pbil.ibcp.fr/cgi-bin/npsa_automat.pl?page=npsa_sopma.html).

### Tertiary structure prediction through homology modeling

Modeller v9.10 [7] was used for predicting tertiary structure and Chimera software was used for displaying different patterns like secondary structure, and physiological properties of protein sequences. PDB Structure 1 F23 was used as a template for homology modeling.

RETRACTED

### Evaluation of homology model

To check the stereochemical quality of the HIV gp41 model, The Procheck suite of programs was used to construct Ramachandaran plot [8] for model validation.

### Phylogenetic analysis

The evolutionary history was inferred using the Neighbor-Joining method [9]. Bootstrap method [10] was used to check the reliability of results. The evolutionary distances were computed using the Poisson correction method [11] and are in the units of the number of amino acid substitutions per site. The analysis involved 9 amino acid sequences. All positions containing gaps and missing data were eliminated. Evolutionary analyses were conducted in MEGA5 [12].

## Results

### Sequence alignment and conservancy

Phylogenetic analysis shows that HIV gp41of Pakistani origin is sharing common ancestry with Russia, China and Uganda while has distant relationship with India and its other neighboring countries (Figure 1a). Three amino acids in the gp41 sequence *i.e.* Threonine, Alanine and Aspartate at positions 13, 22 and 32 respectively are showing most frequent mutations (Figure 1b).

**Figure 1:** HIV gp41 amino acid sequence: a, Phylogenetic Analysis of HIV gp41 Sequences, b, Position 13, 22 and 32 shown in Blue are most frequently mutated gp41amino acids.

### T-cell epitopes of HIV gp41 protein prediction

T-cell epitopes were predicted using Epigen online software on the basis of IC50 value. HLA 0201 showed minimum IC50 value, ensuring maximum binding affinity among all residues (Table 1). Epitopic residues with lowest IC50 predicted values are shown in Figure 2a.

**Table 1:** Predicted T cell epitopes

**T Cell Epitope**			
HLA 0201			
**Starting Position**	**Peptide**	**–logC50 (M)**	**IC50 Value (nM)**
**14**	LLHSLIEEA	9.075	0.84
**7**	EINNYTTLL	8.611	2.45
HLA 0301			
**30**	EQDLLELDK	7.296	50.58
**18**	LIEEAQNQQ	6.854	139.96
A* 1101			
**30**	EQDLLELDK	7.497	31.84
**32**	DLLELDKWA	7.018	95.94
B* 07			
**34**	LELDKWASL	6.934	116.41
**28**	KNEQDLLEL	6.254	557.19

**Figure 2:** a, 3D Model showing Epitopic region of gp41with maximum affinity, b, Tertiary structure of gp41 contains 2 helices.

### Molecular characterization of gp41

Various servers were used to find Glycosylation sites in envelope protein. No such sites were found in gp41 sequence [13-15]. N-glycosylation sites are searched as Asn-X-Ser or Asn-X-Thr sequences, where X is any amino acid residue.

### Secondary and tertiary structure prediction

Secondary structure contains 93.48% helices and 6.52% turns but contains no extended sheets as predicted by SOPMA.

RETRACTED

Tertiary structure of gp41 was constructed using Moeller v 9.10. Chimera was used for model visualization. It was observed that its structure contains 2 helices covering most of the region, and coils but has no Beta pleated sheet (Figure 2b). Using Procheck server Ramachandaran plot was constructed to verify the validity of 3D structure. 93.2% residues were lying in the most favorable region while 6.8% residues were present in additionally allowed region. No residue was observed in generously allowed or disallowed region.

### Phylogenetic analysis

The evolutionary history was inferred using the Neighbor-Joining method [9]. The optimal tree with the sum of branch length = 7.60693736 is shown. The percentage of replicate trees in which the associated taxa clustered together in the bootstrap test (200 replicates) are shown next to the branches [10]. The evolutionary distances were computed using the Poisson correction method [11] and are in the units of the number of amino acid substitutions per site. The analysis involved 9 amino acid sequences. All positions containing gaps and missing data were eliminated. There were a total of 45 positions in the final dataset. Evolutionary analyses were conducted in MEGA5 [12].

## Discussion

In this study 194 sequences were randomly selected from 200 total no of sequences available at the NCBI database. Mutations were observed in all the aligned sequences and it was found that these mutations are more frequent at 3 positions. These amino acid positions are 13, 22 and 32. At position 13, instead of Threonine (T), Serine (S) and Asparagine (N) were observed in most of the cases. Serine (S) was observed instead of Alanine (A) at position 22 in many sequences while instead of Aspartic Acid (D), Glutamic acid (E) was observed at position 32 in many sequences. Mutations were also found at some other positions but these mutations were not frequent and occurred seldom when all the sequences were compared. 1–12 and 33–46 regions were found conserved in all the sequences except two sequences. While two regions, 16–21 and 23–31, were absolutely conserved in all the sequences. Amino acid composition of the sequence was checked and it was observed that Tryptophan is having maximum percentage *i.e.* 204.23% while serine was present in in least amount i. e. 105.09%. Tertiary structure of HIV gp41 was predicted on the basis of homology modeling using MODELLER software. PDB structure 1 F23 was used as a template for homology modeling. HIV gp41 was molecularly characterized using various online servers and it was observed that it has no Glycosylation site or Myrisylation site while it has 0.75% Protein Kinase A sites and 0.58% Casein Kinase 2 Sites. T cell epitopes, A*0201, A*0301, A*1101 and B*07, were predicted using Epijen online software. These epitopes were HLA alleles and have been reported in more than 90% of the world population, regardless of ethnicity. IC50 values were calculated and IC50 value was found least for HLA 0201showing their higher affinity as compared to other alleles. While in rest of the epitopes IC50 value was quite high showing very low affinity.

RETRACTED

Evolutionary relationship was checked among HIV gp41 sequence of various countries. Pakistan and India share common ancestor but this result is not reliable. Very reliable results were obtained that Uganda shares a common ancestor with China, Russia, Africa, Saudi Arab and Afghanistan and also that Africa shares a common ancestry with Saudi Arab and Afghanistan. No reliable results were obtained about the ancestry of HIV gp41 sequence of India, Pakistan and Nigeria.

## Conclusion

The study revealed potential HIV subtype a derived cytotoxic T cell (CTL) epitopes from viral proteome of Pakistani origin. The conserved epitopes are highly useful for the diagnosis of the HIV 1 subtype a. This study will also help scientists to promote research for vaccine development against HIV 1 subtype a to save Pakistani population from potential threats of HIV.

## Competing interest

The authors declare that they have no competing interest.

## Authors’ contribution

SSJ and MS designed the study. MS and SBJ performed the immunoinformatics analysis and rafted the manuscript. SK critically reviewed the manuscript. All authors have read and approved the final manuscript.
